The article "Point Tracking Technology of Sports Image Sequence Marks Based on Fuzzy Clustering Algorithm" was retracted in 2023. Reasons: unreliable results or conclusions; concerns about the data; concerns about the peer review; concerns about the citations.

# Point Tracking Technology of Sports Image Sequence Marks Based on Fuzzy Clustering Algorithm

**DOI:** 10.1155/2022/3814252

**Published:** 2022-04-28

**Authors:** Dengfeng Zhang, Yupeng Li

**Affiliations:** ^1^Shandong Sport University, Jinan 250102, Shandong, China; ^2^College of Physical Education and Health, Linyi University, Linyi 276000, Shandong, China

## Abstract

Fuzzy clustering algorithms have received widespread attention in various fields. Point tracking technology has significant application importance in sports image data analysis. In order to solve the problem of limited tracking performance caused by the fuzzy and rough division of moving image edges, this paper proposes a point tracking technology based on a fuzzy clustering algorithm, which is used for the point tracking of moving image sequence signs. This article analyzes the development status of sports image sequence analysis and processing technology and introduces some basic theories about fuzzy clustering algorithms. On the basis of the fuzzy clustering algorithm, the positioning and tracking of the marker points of the moving image sequence are studied. A series of experiments have proved that the fuzzy clustering algorithm can improve the recognition rate of the landmark points of the moving image. For the detection and tracking of moving targets, the fuzzy clustering algorithm can reach the limit faster under the same number of iterations, and the image noise can be reduced to 60% of the original by 5 iterations. This has excellent development value in application.

## 1. Introduction

Sports is not only a challenge and exploration of human limits in terms of speed, strength, and skills but also reflects the degree of social development and the speed of human progress to a certain extent. It reflects the overall national strength and the degree of social civilization. Nowadays, the importance of the promotion of science and technology in the development of sports has become increasingly prominent. Scientific sports are good for health and vice versa. However, various studies have shown that the field of national fitness is still very lacking in support of scientific fitness technology knowledge. This provides a good opportunity for the implementation of large-scale competitive sports technology transfer and integration into national fitness sports.

As experience-based sports training becomes more and more unable to meet people's needs, people are beginning to use the Internet to obtain better sports learning resources. A large number of sports videos on the Internet provide a good resource for scientific analysis of different sports, and extracting and tracking the moving objects in these videos through better analysis methods is what we need to improve. At present, it is difficult for many moving object segmentation algorithms to achieve good results in sports videos so the segmentation effect and real-time performance are not very ideal. Aiming at the slow speed of segmentation of existing moving objects, the accuracy of segmentation is easily affected by the irregular movement and illumination of the object. The article aims to study the target objects with rich changes in the motion form in the sports video. The paper uses a fuzzy clustering algorithm which is a mathematical rule. They can use it to describe the segmentation interval. This algorithm is derived from the pattern clustering theory. This algorithm was first proposed by Dunn, and it has been developed and improved for a long time. At present, the application of this algorithm in various fields has always been a research hotspot.

With the rapid development of computer intelligence technology, more and more scholars are interested in the application of fuzzy clustering algorithms in the image field [1]. Among them, Verma et al. proposed an improved intuitionistic fuzzy clustering algorithm (IIFCM). It considers local spatial information in an intuitively fuzzy way, preserves image details, is insensitive to noise and does not require any parameter adjustments. It can be applied to the segmentation of brain magnetic resonance (MR) images in computer-aided diagnosis and clinical research [2]. But this method has the problem of poor clustering performance. In order to solve the problem of low efficiency due to complex calculations and poor clustering performance, Chen et al. proposed a histogram-based fuzzy clustering algorithm for color images. Color images of histograms are easier to recognize, making the algorithm more advanced. This method constructs a histogram of the red, green and blue (abbreviation of RGB) components of a given color image. It uses some major valleys identified from the fast peak-valley positioning scheme in each global histogram to perform multi-threshold processing on each component histogram. By applying the histogram merging scheme to the RGB three-component histogram and using some of the main valley values obtained from the fast peak-valley positioning scheme, the new histogram is multithresholded again, and the new histogram is reconstructed so as to achieve the purpose of easily identifying the initialization conditions of the cluster centroids and the number of centroids [3]. However, how to apply these methods to the recognition and tracking of moving targets more efficiently and conveniently requires more research. In order to deal with the complex movement of moving objects, Wang and Sheng proposed an improved algorithm for moving target detection and tracking. It is an improved version of the combination of the FCM algorithm and genetic algorithm. This algorithm is used for target tracking and detection together with the Kalman filter algorithm. Experimental results show that the improved algorithm has greater advantages than other clustering algorithms in terms of optical flow characteristics. Good experimental results have also been achieved in terms of improving the clustering accuracy and calculating more accurate targets and the number of moving vehicles that can be effectively tracked [4]. In order to solve the problem of moving objects lost in the process of moving objects extraction, Lee et al. proposed a clustering algorithm using FCM (Fuzzy C-Means) based on previous research. It is a method of combining separated moving objects into one moving object. This method extracts data from moving objects and counts the moving objects to determine the number of clusters and meet the conditions for executing the FCM clustering algorithm. In the proposed method, the color histogram is extracted from the characteristic information of each moving object, and the histogram is continuously accumulated to avoid being sensitive to noise or changes, and the average value is obtained and stored. Finally, some comparison experiments prove the feasibility and applicability of the proposed algorithm [5]. Object detection and tracking are necessary and challenging activities in multiple PC vision scenarios such as security, motor vehicle navigation, and independent robot navigation. In a study, Mahalingam and Subramoniam proposed an effective method that combines fuzzy ant colony optimization (FACO) with an improved kernel fuzzy C-means algorithm (MKFCM) for object segmentation. The FACO algorithm determines the best initial clustering center for MKFCM, thereby improving all applications of fuzzy clustering. For example, the recommended new method for foreground segmentation in image processing is intelligent and dynamic clustering technology for the segmentation of moving objects. After segmentation, the particle filter method is used for target tracking. Morphological operations help the particle filter to effectively track the object. This method can achieve maximum efficiency for pets and hall monitor videos when using the current algorithm for inspection [6]. Although the bias correction FCM, the spatially constrained FCM, and the adaptive weighted average algorithm have been proved to be robust to the noise of image segmentation using local spatial image information, they also have some disadvantages related to noise sensitivity and poor performance. They are limited to single feature input data (i.e., intensity level features), and their robustness and effectiveness to noise depend to a large extent on the key parameter *α*, and it is difficult to find the best value of *α*. In order to overcome these shortcomings, Memon and Lee propose a generalization of these types of algorithms suitable for clustering *M* feature input data. The proposed generalized FCM clustering algorithm with local information (GFCMLI) not only alleviates the shortcomings of standard FCM but also greatly improves the overall clustering performance. In order to prove the effectiveness, efficiency, and robustness of the GFCMLI algorithm to noise compared with traditional methods, experiments have been conducted on several noisy data and natural/real world images [7]. In order to discover the detailed information contained in infrared images, Yuan et al. proposed an intuitive fuzzy entropy clustering algorithm for image segmentation. The objective function of the intuitionistic fuzzy entropy clustering algorithm is constructed by intuitionistic fuzzy distance and intuitionistic fuzzy entropy based on regularization technology. This method studies the conditions of the intuitionistic fuzzy entropy clustering algorithm. The lagrangian multiplier method is used to calculate the attribution function and centroid, and an iterative algorithm is derived from calculating the Lagrangian multiplier coefficient and attribution degree. Finally, the experimental results prove the ability of the intuitionistic fuzzy entropy clustering algorithm to segment infrared images [8]. Although the above research has optimized the application of fuzzy clustering in the target field from various aspects, the fuzzy clustering algorithm still has the disadvantages of high spatial distortion rate, poor clustering performance, and more complicated methods when it is applied to the target tracking of sports images.

The innovation of this article is as follows: (1) The introduction of fuzzy theory into the point tracking technology of sports images. The fuzzy clustering algorithm is used to visually analyze the moving target in sports training so as to better extract the moving target from the background image and track the target's trajectory. This method realizes automatic fast positioning and tracking of target points in sports images. (2) The fuzzy clustering algorithm is used to achieve the accurate depiction of the motion posture of the target object, and it can conduct better research on sports with rich changes in the shape of the target object in the video.

## 2. Point Tracking of Moving Targets Based on Fuzzy Clustering Algorithm

### 2.1. Fuzzy Clustering Algorithm

#### 2.1.1. Fuzzy Theory

The fuzzy concept in fuzzy theory means that the concept of a certain set used to generalize has an indeterminate or more general nature in meaning, and it can also be said that its extension is unclear—for example, youth and juveniles. Youth are generally younger than adolescents. However, the concept of dividing youth and juveniles by age is uncertain. Fuzzy theory is based on fuzzy sets. The functions used in fuzzy sets are attribute functions, also called attribute functions or fuzzy element functions. Whether an element in a collection belongs to a specific subcollection can be explained by an indicator function. The value of the indicator function of a certain element may be 0 or 1, and the attribute function of this element will be a value between 0 and 1, which indicates the “true degree” of the element belonging to a fuzzy set [9].

Fuzziness can be expressed by the following formula. In the deterministic set, set B is uniquely determined, and the expression is as follows:

(1) $$\begin{array}{c} \chi_{B}\left(y\right)=\left\{\begin{array}{cc} 1 & y\in B,\\ 0 & y\notin B. \end{array}\right. \end{array}$$

That is, one and only one of *y* ∈ *B* and *y* ∉ *B* can be established, whether *y* belongs to set B depends entirely on whether the value of *χ*_*B*_(*y*) is 1. There is a one-to-one mapping relationship between elements and sets, and the boundaries are clear.

The boundaries of fuzzy set theory are vague. In order to describe this theory, the researchers mapped the discrete binary judgments of 0 and 1 in the classical set to the continuous domain [0, 1].

Suppose *T* is the universe of discourse, as a function of *γ*_*B*_ controlling *γ*_*B*_, its value range is [0, 1], namely:

(2) $$\begin{array}{c} \gamma_{B}:T⟶\left[0,1\right],\\ \gamma ⟶\gamma_{B}\left(\gamma \right). \end{array}$$

The attribution function of set *B* is *γ*_*B*_(*γ*), the degree of belonging of element *γ* is affected by the value of *γ*_*B*_(*γ*). The greater the possibility that *γ*_*B*_(*γ*) is close to 1, the higher the degree of belonging of *γ*; the closer *γ*_*B*_(*γ*) is to 0, the lower the degree of membership of *γ* is.

For a discrete finite set *T*={*γ*_1_, *γ*_2_, ..., *γ*_*n*_}, the fuzzy set can be expressed as *B*={*γ*_*B*_(*γ*_1_), *γ*_*B*_(*γ*_2_), ..., *γ*_*B*_(*γ*_*n*_)} [10]. In order to better express the concept of the degree of belonging of the domain elements, Zadeh proposed the following form of expression:

(3) $$\begin{array}{c} B=\sum_{i=1}^{n}\gamma_{B}\frac{\left(\gamma_{i}\right)}{\gamma_{i}}. \end{array}$$

Among them, *γ*_*B*_(*γ*_*i*_) is the degree of attribution of *γ*_*i*_ to *B*. *γ*_*B*_(*γ*_*i*_)/*γ*_*i*_ represents the characteristics of the existence of element *γ*_*i*_ and the attribution function special relationship. This does not mean dividing the numerator by the denominator.

For a continuous set *T*, its fuzzy set can be expressed by (3):

(4) $$\begin{array}{c} B=\int_{\gamma \in T}\frac{\gamma_{B}\left(\gamma \right)}{\gamma }. \end{array}$$

Same as formula (3), *γ*_*B*_(*γ*_*i*_)/*γ*_*i*_ represents the special relationship between element *γ*_*i*_ and the attribution function, and the meaning of “∫” only represents the summarization of each element with its degree of belonging relationship.

#### 2.1.2. Fuzzy Clustering Algorithm

Clustering refers to the process of dividing some similar data into one category and then integrating them into different categories to simplify the data. In the field of mathematical research, the clustering problem can be simply described as follows: There is a d-dimensional data set containing *N* points, denoted as *Rd*, and its cluster number *k* (*k* < *N*) [11]. Fuzzy clustering algorithm is an iterative unsupervised soft clustering method, which comes from pattern clustering theory.

The principle of the fuzzy clustering algorithm is as follows: The objective function is optimized to obtain the membership degree of each sample point to all cluster centers, so as to determine the category of the sample point to achieve the purpose of automatically classifying the sample data. Substitute the image data set *Y*={*y*_1_, *y*_2_, ..., *y*_*n*_} into the objective function iteration to find the minimum value of the function. Thus, the data set is divided into *c* different fuzzy classes. Using (3) to find the cluster centers of each class, using (3) to perform a nonlinear iteration of the objective function to find the extreme points of the objective function, using the objective function (4) to determine the effect of classification, we have the following:

(1) Objective function definition

(5) $$\begin{array}{c} F\left(S,G\right)={\overset{n}{\underset{j=1}{\sum }}\sum_{i=1}^{c}s_{ij}^{l}y_{j}-g_{i}}^{2}. \end{array}$$

In the formula, *n* is the total number of pixels, *c* is the number of clusters. *S* = {*s*_*ij*_} is a matrix of attribution degree, which is used to indicate the attribution degree of voxel *y*_*j*_ in the *i*-th category. *G*={g_1_, g_2_, ..., g_*c*_} is used to represent each cluster center point in the *i*-th category. *l* is an adjustable parameter used to measure the degree of blurring of the segmented result. Attribution function *s*_*ij*_ is used to describe how much voxel *y*_*j*_ belongs to *g*_*i*_ categories.

(2) Constraints of the objective function

(6) $$\begin{array}{c} \overset{c}{\underset{i=1}{\sum }}s_{ij}=1;\;0\leq s_{ij}\leq 1;\;\sum_{j=1}^{n}s_{ij}>0. \end{array}$$

(4) is derived according to the basic idea of the Lagrangian multiplier method and the corresponding constraint (5):

(7) $$\begin{array}{c} G={\overset{n}{\underset{j=1}{\sum }}\sum_{i=1}^{c}\left(s_{ij}^{l}\right)y_{j}-g_{i}}^{2}+\lambda \left(1-\sum_{i=1}^{c}s_{ij}\right). \end{array}$$

The first-order necessary condition of the Lagrangian equation in the optimization formula (7) is as follows:

(8) $$\begin{array}{c} \begin{array}{c} \partial G\\ \partial \lambda \end{array}=1-\overset{C}{\underset{i=1}{\sum }}s_{ij}=0, \end{array}$$

(9) $$\begin{array}{c} \begin{array}{c} \partial G\\ \partial \lambda \end{array}=l{\left(s_{ij}\right)}^{l-1}y_{j}-g_{i}^{2}-\lambda =0. \end{array}$$

From (8):

(10) $$\begin{array}{c} s_{ij}={\left[\begin{array}{c} \lambda \\ \begin{array}{cc} l & y_{j}-g_{i}^{2} \end{array} \end{array}\right]}^{1/\left(l-1\right)}. \end{array}$$

Substituting (9) into (5), we get the following:

(11) $$\begin{array}{c} \overset{c}{\underset{i=1}{\sum }}s_{ij}=\overset{c}{\underset{i=1}{\sum }}{\left(\begin{array}{c} \lambda \\ l \end{array}\right)}^{1/\left(l-1\right)}{\left[\begin{array}{c} \lambda \\ y_{j}-g_{i}^{2} \end{array}\right]}^{1/\left(l-1\right)}\\ ={\left(\begin{array}{c} \lambda \\ l \end{array}\right)}^{1/\left(l-1\right)}\left\{\sum_{i=1}^{c}{\left[\begin{array}{c} \lambda \\ y_{j}-g_{i}^{2} \end{array}\right]}^{1/\left(l-1\right)}\right\}\\ =1 \end{array}$$

Thus,

(12) $$\begin{array}{c} \lambda^{1/\left(l-1\right)}={\sum_{k=1}^{c}\left[\begin{array}{cc} l & y_{j}-g_{i}^{2} \end{array}\right]}^{1/\left(l-1\right)}. \end{array}$$

Substituting the above formula into (10), we can get the following:

(13) $$\begin{array}{c} s_{ij}=\frac{1}{\left\{\sum_{k=1}^{c}{\left[\begin{array}{c} y_{j}-g_{i}\\ y_{j}-g_{k} \end{array}\right]}^{21/\left(l-1\right)}\right\}}. \end{array}$$

(3) Attribution function of the objective function

A series of derivations of (4) according to the principle of the Lagrangian multiplier method and corresponding constraint (5), the attribution function of the objective function is obtained as follows:

(14) $$\begin{array}{c} s_{ij}=\begin{array}{c} y_{j}-g_{i}^{-2/\left(l-1\right)}\\ \overset{c}{\underset{k=1}{\sum }}y_{j}-g_{k}^{-2/\left(l-1\right)} \end{array}. \end{array}$$

In the same way, if the partial derivative of *g*_*i*_ is obtained and then the terms are further shifted, the obtained attribution degree and the expression of the cluster center are as follows:

(15) $$\begin{array}{c} g_{i}=\begin{array}{c} \overset{n}{\underset{j=1}{\sum }}s_{ij}^{l}y_{j}\\ \overset{n}{\underset{j=1}{\sum }}s_{ij}^{l} \end{array}. \end{array}$$

According to the classification number of the sample data set, the fuzzy clustering algorithm uses (13) and (14) to determine the attribution matrix and cluster center of the sample. It is achieved by repeatedly iteratively optimizing the objective function (4), and the specific steps are as follows:

  Step 1: Set the cluster center *G*0 {*g*1, *g*2,…, *gc*} and initialize the attribute matrix *S*0, determine the values of *c* and *l*, determine the iteration stop judgment value *l* > 0, and initialize the number of iterations *k* > 0.
  Step 2: Derive the belonging degree matrix *Sk* by (6) and the class center point matrix.
  Step 3: Use *Sk* to update the cluster center matrix *Gk* according to (6).
  Step 4: If *G*' (*k* + 1) > *G'* (*k*), the algorithm stops. Otherwise, repeat steps 2 and 3, and set *k* = *k* + 1.

### 2.2. Detection and Segmentation Methods of Moving Targets

#### 2.2.1. Moving Target Detection

There are many commonly used methods for moving target detection, one of which is the frame difference method. Since the images of consecutive frames in a video sequence are different, target detection and extraction can be performed based on this difference. Since the images of consecutive frames in a video sequence are different, target detection and extraction can be performed based on this difference. It also uses an image threshold segmentation method, mainly through pixel time difference and image binarization, to extract moving targets [12]. Image threshold segmentation is image binarization, which is to set a threshold *T*, a group of pixels larger than *T* and a group of pixels smaller than *T*. It sets the gray value of the pixels on the image to 0 or 255, which means that the entire image presents an obvious visual effect of only black and white.

The mathematical expression formula of the three-frame difference method is as follows:

(16) $$\begin{array}{c} w_{t}\left(i,j\right)=\left|p_{t-1}\left(i,j\right)-p_{t}\left(i,j\right)\right|\times \left|p_{t}\left(i,j\right)-p_{t+1}\left(i,j\right)\right|,\\ W_{t}\left(i,j\right)=\left\{\begin{array}{c} 255,w_{t}\left(i,j\right)>T,\\ 0. \end{array}\right. \end{array}$$

Among them, *p*_*t*−1_(*i*, *j*) is the first frame of the three-frame difference method image, *p*_*t*_(*i*, *j*) is the second frame, *p*_*t*+1_(*i*, *j*) is the third frame, *w*_*t*_(*i*, *j*) is the three-frame changing part of the image. After selecting the appropriate threshold T, the target object is directly extracted from the multivalue digital image. *W*_*t*_(*i*, *j*) is the binary image of the moving target in the middle frame [13].

The three-frame difference algorithm is an improved method of the adjacent two-frame difference algorithm. It selects three consecutive frames of video images for difference operation to eliminate the influence of the exposed background due to motion, thereby extracting accurate contour information of the moving target.

The algorithm of the three-frame difference method is simple, does not consider the background information, and its shortcomings are also obvious. This algorithm has higher requirements on the number of received frames and the target speed. If the target moves very fast and the selection time is long, it is more difficult to form a coverage area and cannot be formed between frames. As a result, the moving target cannot be divided. Conversely, if the moving target is too slow and the time between selected frames is short, it will cause the target to overshoot and make the target look like something hollow. Even if the object is completely covered, it is impossible to find a moving target.

*(1). Image Segmentation Evaluation Standard.* In order to quantitatively evaluate the clustering results of the algorithm, this paper uses the segmentation coefficient (*v pc*) and the segmentation entropy (*v pe*) to give two evaluation indicators.

(1) Division coefficient *zpc*
  (17) $$\begin{array}{c} z_{pc}\left(S\right)=\begin{array}{c} 1\\ n \end{array}\sum_{j=1}^{n}\overset{c}{\underset{i=1}{\sum }}s_{ij}^{2}. \end{array}$$
(2) Division coefficient *zpe*
  (18) $$\begin{array}{c} z_{pe}\left(S\right)=-\begin{array}{c} 1\\ n \end{array}\sum_{j=1}^{n}\overset{c}{\underset{i=1}{\sum }}s_{ij}\mathrm{lg}s_{ij}. \end{array}$$

In formula (19), *n* is the total number of pixels, *c* is the number of clusters, and *s*_*ij*_ is the attribute function in fuzzy clustering. For fuzzy sample sets, the samples should be continuous and closed, and each sampling point has a unique classification [14]. The value range of the division coefficient *zpc* is 1/*c*, 1. In the determined range, the higher the index value, the better the clustering effect. That is to say, the closer the *zpc* value is to 1, the clearer the clustering result will be; the closer the *zpc* value is to 1/*c*, the less clear the clustering result. *zpe* is the segmentation entropy. The lower the index value in a certain range, the better the clustering effect, and the best clustering effect is obtained when the minimum value is reached.

In addition, this paper uses the manual segmentation results as the standard to evaluate the segmentation results of the algorithm using Segmentation Accuracy (*SA*). The definition of segmentation accuracy is shown in (18):

(19) $$\begin{array}{c} SA=\frac{\text{Number of pixels correctly classified}}{\text{Total number of pixels}}\times 100\%. \end{array}$$

In (18), the numerator is the number of correctly classified pixels, and the denominator is the number of all pixels.

#### 2.2.2. Single Target Segmentation

In some sports occasions, there is only one person as the subject of the exercise, such as rock climbing, shooting, gymnastics, etc. In this case, the camera lens only tracks a single subject, or only focuses on a fixed target. Or in the presence of other moving subjects, the lens also only needs to track a moving target in a complex environment (there are many objects in the environment and the background is more complicated). Therefore, it is only necessary to detect when the target is in motion only in the camera lens, and the target segmentation method at this time is relatively easy. Using the information of the image as a whole, or using the available information from the part of the image, select the appropriate threshold and determine the pixel attribution by comparing the gray value of the pixel with the threshold [15]. Single threshold sets a threshold, that is, a gray value divides the image into two categories, and multithreshold sets multiple different gray values as thresholds for segmentation. The image can be divided into multiple different areas so as to distinguish the available target area in the image and the background area that needs to be eliminated.

#### 2.2.3. Multitarget Segmentation

In other sports, such as football, basketball, volleyball, rugby, marathon, and other multiplayer sports, there will be multiple sports targets in the field of view of the photographic equipment at the same time. Cluster analysis has obvious advantages in this case. Image segmentation is essentially a problem of pixel clustering. In complex scenes, multiple moving targets will have inaccurate clustering, and the advantage of the fuzzy clustering algorithm is to achieve better classification in situations involving fuzzy boundaries [16].

The first step is to mark multiple moving targets. The purpose of marking is to distinguish different targets. In the marking process, because the connectivity of the binary image is not necessarily ideal, the same motion can be combined together, that is, using two or more network markings, and some isolated noise points may be marked with numbers. Therefore, it is also necessary to detect the area and distance of the marked target. This step is also very important for removing targets with smaller surface areas and merging targets that are closer to each other. Then, the targets marked with different numbers are processed separately to find the smallest circumscribed rectangle and use this to represent the target.

### 2.3. Moving Target Tracking

The so-called target tracking is that we first detect the image where the target is located and then obtain the motion parameters and motion trajectory of the moving target through the comparison and analysis of the moving image sequence. The effective features of the moving target are obtained by comparison, analysis, and detection. At this time, we use appropriate tracking algorithms to find available candidate regions near the moving target in the image. The variability of this candidate region is relatively large in a short time. Therefore, this area can be used as a new standard target to determine the correlation of the next frame [17]. In practical applications, the results of target monitoring can be used to detect target speed, describe motion trajectories, flow detection, and other purposes, understand the behavior of moving targets, or complete more advanced work. Moving target monitoring methods mainly include matching target-based methods, model-based methods, attributes and characteristics-based monitoring methods, and chart-based monitoring methods. Among them, the standard matching method uses grayscale or correlation or similarity between images as the basis for judgment. The basic composition is shown in Figure 1.

As can be seen from Figure 1, the complete moving target detection and tracking process mainly includes four parts. The first part is a video capture device, the second part is motion area detection, the third part is target feature extraction, and the fourth part is target tracking. And this motion tracking system can be subdivided into the steps shown in Figure 2:

Moving target detection and tracking are mainly to combine the detection and tracking, and the image processing of the detection part should make the later tracking easier. First, the camera captures the color video images that need to be analyzed and then converts the acquired image sequence through grayscale. The next step is to sharpen the grayscale converted image. Next, the motion area is approximately detected by the method of frame difference or background difference. Finally, perform binarization, filtering, and morphological processing on the detected areas, respectively. Determining the target feature value and using various tracking algorithms to track subsequent frames. In the tracking process, in order to reduce the amount of calculation, the possible location of the target can be estimated [18].

## 3. Point Tracking Experiment and Analysis of Sports Image Sequence Signs

### 3.1. Sports Image Segmentation under Fuzzy Clustering Algorithm

This experiment used the final video of the 2020 Volleyball Championship as the object. A segment of continuously changing moving images is selected from the first half and the second half for segmentation, and the spatial accuracy of each segmentation method is evaluated by (16).

Under normal circumstances, in a segmentation method, the smaller the SA value, the higher the spatial accuracy of this method.

The SA calculation results are shown in Table 1. The SA value of the fuzzy clustering algorithm used in this article is lower than the other three algorithms. The spatial precision of segment 1 is lower than that of segment 2, which may be because segment 1 has a simpler background than segment 2 and is less difficult to segment. From the experimental results, it can be seen that the fuzzy clustering algorithm can effectively fill the gap in the sports video space and avoid the vacancy in the image segmentation area. Even in the face of images with more complex environments and colors, it can still be segmented more accurately, and the spatial accuracy is higher than that of ordinary methods [19].

#### 3.1.1. Noise Iteration Performance

Noise is meaningless data, which has always been a difficult point in the field of image segmentation. Many methods are sensitive to noise, so for a clearer and more accurate image. The segmentation method needs to get rid of the interference of irrelevant data as much as possible, so the segmentation method needs to perform noise iteration on the segmented image. If the data contains a lot of meaningless data, it will affect the convergence speed of the data, so the most important part of noise iteration is to speed up the convergence speed. In Figure 3, the noise of segment 1 is generally higher than that of segment.

Figure 4 is the correlation curve between the number of iterations.

In Figure 4, under the processing of four different segmentation methods, the image noise of segment 1 and segment 2 are all reduced. But in terms of convergence speed, the FCA is obviously better. Under the same number of iterations, the FCA can reach the limit faster. 5 iterations can reduce the image noise to 60% of the original, and it has better noise iteration capability than other methods.

It can be seen from Figure 4 that the experiment compares MPEG-4, frequency domain segmentation, and time domain segmentation. Segmentation of sports images with the same degree of noise superimposed to verify the accuracy and stability of the fuzzy clustering algorithm. The comparison shows that the fuzzy clustering algorithm is better in noise processing than the other three methods [20].

### 3.2. Realization of Tracking and Positioning under Fuzzy Clustering Algorithm

In order to verify the effect of the algorithm, this paper conducts a table tennis game video tracking simulation experiment on the MATLAB platform. The tracking result of the table tennis game video is shown in Figure 5.

Figure 5 shows the six frames extracted from the tracking result of the player's serve video in a table tennis match.

### 3.3. Single-Sensor Multitarget Tracking

This paper conducts a table tennis game video tracking simulation experiment on the MATLAB platform. The tracking result of the table tennis game video is shown in Figure 5.

It can be seen from Figure 6 that there will still be tracking divergence when using traditional algorithms. The tracking result of a single sensor is improved by FCA. When the sensor is used to track the target and when the target is very close, the traditional algorithm is easy to produce correlation errors and cause the divergence of the target tracking, and the target will be lost after a long time.

FCA overcomes the shortcomings of traditional algorithms.  Table 2 shows the average tracking error of the two algorithms. It can be seen that the FCA can obtain better tracking results than traditional algorithms.

## 4. Discussion

This article first introduces the fuzzy theory and its concept of the collection, then focuses on the theory of FCA and its algorithm steps in image segmentation, and shows the derivation process of the fuzzy clustering principle. This paper proposes a sports target tracking method based on fuzzy clustering. In this method, the degree of attribution is used as a weighting factor. After weighing the amount of information with the weighting factor, this information amount is regarded as the total information amount of the target at a certain time. The traditional algorithm only selects one measuring point trajectory for each target as the echo target, ignoring the certainty and uncertainty of information caused by noise and interference. Therefore, when the targets are dense, it is easy to cause correlation errors, leading to tracking deviation. The algorithm reduces the certainty and uncertainty of information through the weighting process, thereby ensuring the monitoring of multiple high-precision targets.

FCA has the advantages of strong local search ability, simpler application method, simple design and fast calculation speed. However, due to its inherent shortcomings, traditional fuzzy grouping algorithms have encountered great problems when implementing image segmentation. In order to overcome the problems faced by traditional fuzzy clustering methods in the field of image segmentation, researchers have done a lot of work to improve. In this paper, the FCA itself is improved, and the improved algorithm is applied to image segmentation in order to obtain a better segmentation effect and expand the range of feature extraction of the FCA.

FCA derives the image sequence from the motion video playback state and predicts and compensates for the motion of the target object according to the order of the pictures. Creating the same background in many images with a short distance from each other, exporting time-domain difference images from adjacent image frames with different frame values, defining unclear features when moving the target object, and writing the corresponding performance function.

In order to verify the effectiveness and accuracy of the FCA in this paper, a video tracking simulation experiment of a table tennis game and a comparison experiment of single-sensor multi-target tracking are carried out. In a complex environment with large background interference, feature points are extracted from sports pictures and athletes are matched. It can be seen that in the complex sports environment, the algorithm in this paper can effectively calculate and reduce the extraction of wrong feature points. Whether in the extraction of feature points or the matching of moving targets, the performance is better than traditional algorithms.

## 5. Conclusions

In this paper, we use this method of analyzing sports video images to track sports goals is helpful to understand the technical laws of different sports and the characteristics of different people's fitness. Providing better professional services for professional sports curriculum education improves the level of competitive sports athletes and the national recreation and fitness. In the simulation experiment, the application of the fuzzy algorithm on the sports video has achieved relatively satisfactory results. In terms of real-time performance, the algorithm does not involve complex mathematical operations. Compared with existing methods, it has certain advantages in computing speed and can meet real-time requirements. With comprehensive consideration of various indicators, the FCA is a robust and efficient sports image analysis algorithm.

## Figures and Tables

**Figure 1:** Basic composition diagram of moving target tracking.

**Figure 2:** Schematic diagram of moving target detection and tracking.

**Figure 3:** Image noise average curve.

**Figure 4:** The relationship between the number of iterations of segment 1 and segment 2 and the average value of noise.

**Figure 5:** Target tracking result of a table tennis match.

**Figure 6:** Multitarget tracking results under the two algorithms.

**Table 1:** Statistics of SA values.

Segmentation method	Segment 1	Segment 2
FCM	0.0814	0.2255
MPEG-4	0.1529	0.3164
Time domain segmentation (TDS)	0.1661	0.4591
Frequency domain segmentation (FDS)	0.2819	0.3651

**Table 2:** Average tracking error/m of the two algorithms.

Target	FCM	Traditional algorithm
Target 1	19.6297	27.3206
Target 2	17.6898	28.4696

## Data Availability

No data was used to support this study.
